The article "The Impact of Intraoperative Imaging on Outcomes in Combined Neurosurgical and Reconstructive Procedures: A Systematic Review" was retracted in 2025. Reasons: unreliable results or conclusions; concerns about the authorship.

# The Impact of Intraoperative Imaging on Outcomes in Combined Neurosurgical and Reconstructive Procedures: A Systematic Review

**DOI:** 10.7759/cureus.86035

**Published:** 2025-06-15

**Authors:** Muhammad Ilyas Alozai, Omar Amgad Yehia Elassra, Aliaa H Alkhazendar, Ahmed S Ibrahim, Abdul Sattar Gatta, Syed Muhammad Baqar Raza, Abdelrahman Sahnon Abaker Sahnon, Jarallah HJ Alkhazendar, David O Oriko, Shafaq Mushtaq

**Affiliations:** 1 Internal Medicine, Punjab Medical College, Faisalabad Medical University, Faisalabad, PAK; 2 Emergency Medicine, North Manchester General Hospital, Manchester, GBR; 3 Plastic Surgery, Ain Shams University, Cairo, EGY; 4 Surgery, The Islamic University of Gaza, Gaza, PSE; 5 Orthopedics and Traumatology, Royal Care International Hospital, Khartoum, SDN; 6 Accident and Emergency, Liaquat National Hospital, Karachi, PAK; 7 Medicine, Liaquat College of Medicine and Dentistry, Jinnah Sindh Medical University, Karachi, PAK; 8 Cardiac Surgery, Rawalpindi Institute of Cardiology, Rawalpindi, PAK; 9 Vascular Surgery, Evangelisches Krankenhaus Hubertus, Berlin, DEU; 10 General Physician, Speedy Recovery Clinic, Jeddah, SAU; 11 General and Emergency Surgery, East and North Hertfordshire NHS Trust - Lister Hospital, Stevenage, GBR; 12 Neurology, University of Maryland Medical Center, Baltimore, USA; 13 Surgery, Liaquat National Hospital, Karachi, PAK

**Keywords:** clinical trials, imri, intraoperative imaging, intraoperative ultrasound, neuronavigation, neurosurgery, reconstructive surgery, surgical outcomes

## Abstract

This systematic review evaluates the impact of intraoperative imaging on surgical outcomes in combined neurosurgical and reconstructive procedures. A comprehensive literature search was conducted across four databases, including PubMed, Scopus, Web of Science, and the Cochrane Central Register of Controlled Trials (CENTRAL), focusing on clinical trials published between 2019 and 2024. Following Preferred Reporting Items for Systematic Reviews and Meta-Analyses (PRISMA) guidelines, six studies that met stringent eligibility criteria were selected, including randomized controlled trials (RCTs) and prospective cohort studies involving imaging modalities such as intraoperative MRI (iMRI), intraoperative ultrasound (iUS), fluoroscopy, neuronavigation, and machine vision-based systems. Data were extracted on sample size, intervention type, control group characteristics, and primary surgical outcomes, including extent of resection, complication rates, and functional recovery. Qualitative synthesis revealed consistent benefits associated with intraoperative imaging, including enhanced anatomical precision, reduced complication rates, improved extent of resection, and fewer reoperations. Quality appraisal indicated low to moderate risk of bias across most studies. These findings endorse the broader integration of intraoperative imaging into complex surgical workflows and highlight the need for further research in reconstructive domains.

## Introduction and background

Advancements in surgical techniques over recent decades have brought forth a growing reliance on intraoperative imaging technologies to enhance precision, safety, and patient outcomes [1]. Among the many fields benefiting from these innovations, neurosurgery stands out due to the intricacy of anatomical structures and the critical need for preserving functional tissue. Intraoperative imaging modalities such as intraoperative MRI (iMRI), intraoperative ultrasound (iUS), fluoroscopy, and fluorescence-guided techniques have emerged as indispensable tools in facilitating real-time navigation and improving surgical accuracy during complex cranial and spinal procedures [2]. These modalities enable surgeons to visualize anatomical details with heightened clarity, enabling more complete tumor resections, reduced operative complications, and enhanced neurological outcomes. Simultaneously, reconstructive surgery, especially when performed in conjunction with neurosurgical procedures, demands a similarly high level of precision [3].

Whether in the context of skull base tumor resections, craniofacial trauma, or peripheral nerve repairs, intraoperative imaging supports surgeons in achieving both functional and aesthetic goals while minimizing iatrogenic injury. The integration of imaging during reconstructive phases has been shown to reduce reoperation rates, improve graft or flap placement, and assist in preserving neurovascular structures [4]. However, while the individual benefits of intraoperative imaging in neurosurgery and reconstructive surgery are well documented, literature remains sparse when it comes to systematically evaluating its role in combined neurosurgical and reconstructive procedures, a scenario where precision, coordination, and intraoperative decision-making are especially critical.

Recent clinical trials have begun to explore the outcomes associated with intraoperative imaging in various surgical specialties. Emerging evidence supports its role in reducing complications, increasing the extent of tumor resections, decreasing operative times, and improving long-term functional recovery. Nevertheless, a consolidated evaluation of its effectiveness in multidisciplinary surgeries, where both neurosurgical and reconstructive components are involved, is lacking. Understanding the true impact of these imaging techniques in such integrated procedures is essential for developing evidence-based guidelines, optimizing resource allocation, and ultimately improving patient care.

In light of this, the objective of this systematic review is to evaluate the clinical impact of intraoperative imaging modalities on surgical outcomes in procedures that involve both neurosurgical and reconstructive elements, by using the PICO (Population, Intervention, Outcome measures) framework [5]: Population includes patients undergoing combined neurosurgical and reconstructive surgeries; Intervention refers to the use of intraoperative imaging (e.g., MRI, ultrasound, fluoroscopy, fluorescence); Comparison is with surgeries performed without such imaging; and Outcomes include surgical precision, extent of resection, complication rates, reoperation rates, and functional recovery. This review aims to synthesize evidence from recent clinical trials (within the last five years) to assess the utility and effectiveness of intraoperative imaging in this high-stakes surgical domain.

## Review

Materials and methods

Search Strategy

A comprehensive literature search was conducted per Preferred Reporting Items for Systematic Reviews and Meta-Analyses (PRISMA) 2020 guidelines [6]. Databases including PubMed, Scopus, Web of Science, and Cochrane Central Register of Controlled Trials (CENTRAL) were systematically searched. The search focused on clinical trials published in the last five years (2019-2024), using a combination of keywords and Boolean operators such as "intraoperative imaging," "neurosurgical procedures," "reconstructive surgery," "ultrasound," "MRI," "fluoroscopy," "neuronavigation," and "clinical outcomes." Search results were exported into reference management software, and duplicates were removed before screening. Additional manual searches of reference lists were conducted to ensure comprehensive inclusion of relevant studies.

Eligibility Criteria

Studies were selected based on predefined inclusion and exclusion criteria. Inclusion criteria comprised prospective clinical trials, either randomized controlled trials or comparative cohort studies, that explicitly evaluated the use of intraoperative imaging modalities such as iMRI, iUS, fluoroscopy, neuronavigation, or fluorescence-guided imaging. Eligible studies had to involve neurosurgical, reconstructive, or combined neurosurgical-reconstructive procedures and report at least one quantitative surgical outcome, such as extent of resection, complication rate, reoperation rate, operative time, or functional recovery [e.g., deterioration-free survival (DFS) or modified Rankin scale]. Only peer-reviewed articles published in English between 2019 and 2024 were included. Exclusion criteria included non-clinical studies (e.g., in vitro or animal models), case reports, editorials, narrative or systematic reviews, and studies that either lacked outcome data or did not use intraoperative imaging as a primary intervention.

Data Extraction

Data were independently extracted from the final set of included studies using a standardized extraction sheet. Extracted variables included study title, author, year of publication, imaging modality used, study design, sample size, intervention and control group descriptions, outcomes measured, and key findings. Special attention was given to quantitative outcomes such as rates of gross total resection (GTR), progression-free survival (PFS), operative time, radiation exposure, complication rates, and reoperation rates. Any discrepancies in data extraction were resolved through discussion and consensus.

Data Analysis and Synthesis

Due to heterogeneity in imaging modalities, surgical procedures, and outcome measures across studies, a qualitative synthesis was performed. Results from individual trials were organized into comparative tables, enabling cross-study analysis of trends in effectiveness and safety outcomes. No formal meta-analysis was conducted due to variability in methodologies and endpoints. A risk of bias assessment was applied to each study using tools appropriate to the study design: the Cochrane Risk of Bias 2.0 (RoB 2) [7] for randomized controlled trials, Risk of Bias in Non-Randomized Studies - of Interventions (ROBINS-I) for non-randomized comparative studies [8], and the National Institute of Health (NIH) Quality Assessment Tool [9] for single-arm trials. Findings were narratively synthesized to highlight the clinical utility and limitations of intraoperative imaging in enhancing surgical outcomes.

Results

Study Selection Process

The study selection process is outlined in Figure 1, which illustrates the PRISMA 2020 flow diagram. A total of 387 records were identified through four major databases: PubMed (n = 148), Scopus (n = 104), Web of Science (n = 85), and CENTRAL (n = 50). After removing 54 duplicate records, 333 unique studies were screened based on titles and abstracts. From these, 140 were excluded for not meeting the preliminary criteria. Of the 193 full-text reports sought for retrieval, 97 could not be retrieved due to access limitations or incomplete records. Among the 96 full-text reports assessed for eligibility, 90 were excluded for reasons including being reviews or editorials (n = 22), case reports (n = 15), in vitro or animal studies (n = 12), lacking clear outcome reporting (n = 18), or not involving intraoperative imaging as a core intervention (n = 23). Ultimately, six studies met all eligibility criteria and were included in the final qualitative synthesis

**Figure 1:** PRISMA flow diagram depicting the study selection process PRISMA: Preferred Reporting Items for Systematic Reviews and Meta-Analyses

Characteristics of the Included Studies

As detailed in Table 1, the six selected studies encompass a diverse range of intraoperative imaging modalities and clinical contexts within neurosurgical and reconstructive procedures. The imaging techniques evaluated include iUS, diffusion tensor imaging (DTI), iMRI, fluoroscopy, fluorescence-guided surgery, and advanced machine vision-based navigation systems. Study designs primarily consisted of randomized controlled trials, with one phase 1 single-arm study and one comparative cohort study. Sample sizes ranged from 29 to 357 participants, reflecting a mix of exploratory and large-scale evaluations. The outcomes measured were similarly varied, including DFS, GTR, PFS, complication rates, and technical accuracy metrics such as pedicle screw placement. Across studies, the use of intraoperative imaging consistently contributed to improved surgical precision, fewer complications, enhanced functional outcomes, and greater resection rates, underscoring its value in optimizing surgical results in complex anatomical environments.

**Table 1:** Characteristics of the included studies 5-ALA: 5-aminolevulinic acid; DFS: deterioration-free survivall; DTI: diffusion tensor imaging; EBL: estimated blood loss; EGFR: epidermal growth factor receptor; FLASH: fast anatomic scan and high-accuracy navigation; GTR: gross total resection; iMRI: intraoperative magnetic resonance imaging; IOF: intraoperative fluoroscopy; iUS: intraoperative ultrasound; MIS: minimally invasive surgery; mRS: modified Rankin scale; OS: overall survival; PFS: progression-free survival; RCT: randomized controlled trial

Study	Imaging modality sed	Study design	Sample size	Intervention group	Control group	Outcomes measured	Key findings
Plaha et al., 2022 [10]	iUS + DTI	Two-stage RCT	357	Standard surgery + iUS + DTI	Standard surgery with 5-ALA and neuronavigation	DFS	iUS and DTI evaluated for impact on DFS; designed to improve quality of life and disease progression metrics
Li et al., 2024 [11]	iMRI	RCT	321	iMRI-guided glioma resection	Conventional neuronavigation	GTR, PFS, OS, safety	iMRI significantly increased GTR (83.85% vs. 50%) and improved PFS and OS in HGGs, especially in eloquent brain regions
Zhou et al., 2021 [12]	EGFR-targeted fluorescence Imaging (panitumumab-IRDye800)	Phase 1 clinical trial	29	Fluorescence-guided glioma resection	None (single-arm study)	Tumor visualization, extent of resection, and detection of occult tumor	Demonstrated feasibility; improved tumor margin detection and surgical precision
Andrades et al., 2021 [13]	IOF	Comparative cohort study (prospective vs. historical)	100 (49 IOF, 51 non-IOF)	Facial fracture repair with IOF	Facial fracture repair without IOF	Postoperative complications, reoperation rate	The IOF group had fewer complications (2.04% vs. 15.69%) and no reoperations compared to 11.76% in the non-IOF group
Yan et al., 2024 [14]	Neuronavigation-assisted stereotactic drilling	RCT	67	Minimally invasive stereotactic drainage with neuronavigation	Conventional craniotomy hematoma removal	Surgery duration, bleeding volume, ICU stay, complications, mRS at 90 days	The MIS group had shorter surgeries, less bleeding, fewer complications, and better functional outcomes
Malham and Munday, 2022 [15]	FLASH navigation (machine vision) vs. 3D fluoroscopy	Randomized prospective comparative cohort study	90 patients (429 pedicle screws)	FLASH navigation-guided lumbar fusion	3D fluoroscopy-guided lumbar fusion	Radiation time and dose, Pedicle screw accuracy, EBL, Revision rate	FLASH reduced radiation (97.8%), maintained high screw accuracy, and avoided reoperation; practical and efficient alternative to 3D fluoroscopy

Quality Assessment

The quality assessment of the included studies, as presented in Table 2, demonstrated a generally high level of methodological robustness across the selected clinical trials. Of the six studies analyzed, four were RCTs evaluated using the Cochrane RoB 2 tool. These studies were rated as having a low risk of bias, owing to well-structured randomization processes, clearly defined outcomes, pre-registered protocols, and appropriate analytical methods. One RCT with a comparative cohort design was assessed as having low to moderate risk, primarily due to minor baseline imbalances that could introduce selection bias, although outcome measures were rigorously reported. The non-randomized comparative cohort study was evaluated using the ROBINS-I tool and demonstrated a moderate risk of bias, largely due to reliance on a historical control group. Additionally, the phase I single-arm trial was assessed with the NIH Quality Assessment Tool and received a fair rating, reflecting limitations such as the absence of a control group and a small sample size, despite its well-defined objectives and clear reporting. Overall, the quality assessment affirms the reliability of the evidence while identifying key methodological considerations.

**Table 2:** The quality assessment of the included studies NIH: National Institute of Health; RCT: randomized controlled trial; RoB 2: Risk of Bias 2.0 tool; ROBINS-I: Risk of Bias in Non-Randomized Studies - of Interventions

Study	Study type	Tool used	Overall risk of bias	Key comments
Plaha et al., 2022 [10]	RCT (two-stage)	RoB 2	Low	Randomization ii clear, pre-registered protocol, appropriate outcomes, and no major concerns
Li et al., 2024 [11]	RCT	RoB 2	Low	Strong methodology, balanced arms, well-reported outcomes, and appropriate statistical analysis
Zhou et al., 2021 [12]	Phase I, single-arm trial	NIH Tool	Fair	No control group, small sample, but clear objectives and robust reporting for feasibility assessment
Andrades et al., 2021 [13]	Non-randomized comparative cohort	ROBINS-I	Moderate	Historical control introduces bias risk; the prospective arm was well conducted, with meaningful outcomes
Yan et al., 2024 [14]	RCT	RoB 2	Low	Good randomization, clear endpoints, blinded outcome assessment, and low attrition
Malham and Munday, 2022 [15]	RCT (comparative cohort RCT)	RoB 2	Low to Moderate	Randomization adequate; possible selection bias due to baseline imbalance; well-measured outcomes

Discussion

This systematic review of six clinical trials demonstrates that the incorporation of intraoperative imaging modalities such as iMRI, iUS, fluoroscopy, and neuronavigation consistently enhances surgical precision, improves resection outcomes, and reduces complication and reoperation rates in neurosurgical and reconstructive procedures. For instance, Li et al. [11] reported a GTR rate of 83.85% using iMRI vs. 50% with conventional neuronavigation (p<0.0001). Similarly, Andrades et al. [13] found a reduction in bone-related complication rates from 15.69% to 2.04% and a complete elimination of reoperations when fluoroscopy was used in facial fracture surgery. These findings underscore the tangible benefits of real-time imaging in optimizing patient outcomes, particularly in anatomically complex or functionally sensitive surgical regions.

The findings of this review align with prior literature emphasizing the role of intraoperative imaging in enhancing surgical outcomes, especially in neuro-oncology and spinal procedures [16]. Previous systematic reviews have reported GTR rates increasing by up to 30% with iMRI and similar improvements with iUS in glioma surgery. However, many earlier studies lacked rigorous randomization or were limited by observational designs. This review strengthens the evidence base by focusing exclusively on recent clinical trials and expanding the scope to include reconstructive elements. The outcomes observed not only reaffirm current trends toward image-assisted surgery but also reveal an underexplored intersection between neurosurgery and reconstructive disciplines that warrants more structured investigation.

The integration of intraoperative imaging into surgical workflows has the potential to significantly influence preoperative planning, intraoperative decision-making, and interdisciplinary collaboration. For example, the ability to visualize critical neurovascular structures in real-time through DTI and iUS can guide safe tumor resection while preserving function. The reduction of fluoroscopy-related radiation exposure by up to 97.8% using machine vision systems (Malham et al., [15]) not only enhances safety but also supports a shift toward radiation-sparing strategies. These findings suggest that training curricula for neurosurgeons and reconstructive surgeons should incorporate proficiency in advanced intraoperative imaging modalities. Furthermore, institutions may need to reallocate resources toward acquiring and maintaining such imaging systems to align with evolving standards of care. 

Intraoperative imaging enhances surgical outcomes through multiple well-documented mechanisms. It improves anatomical visualization, enabling real-time updates that account for tissue shifts or resections, which is particularly vital in brain and craniofacial surgeries. Techniques such as iMRI and neuronavigation provide precise spatial orientation, facilitating safer dissection around eloquent cortex or cranial nerves [17]. iUS and fluoroscopy enable the surgeon to detect residual pathology or misaligned fractures instantly, allowing corrections before wound closure. This immediate feedback loop directly contributes to reduced reoperation rates and fewer postoperative complications, as seen in the Andrades et al. and Yan et al. trials. In essence, intraoperative imaging functions as a dynamic extension of surgical judgment and precision.

Strengths

A key strength of this review is its methodological rigor, adhering to PRISMA guidelines [6] and employing structured quality appraisal tools such as RoB 2 [7] and ROBINS-I [8]. The inclusion criteria were deliberately stringent, selecting only clinical trials published in the past five years, which ensures that findings reflect contemporary surgical techniques and technologies. Notably, the review bridges a critical gap by focusing on combined neurosurgical and reconstructive procedures, a domain where the interplay between functional preservation and anatomical restoration demands the highest surgical accuracy. This multidisciplinary lens adds both novelty and clinical relevance to the existing body of evidence.

Limitations

Despite its strengths, this review has several limitations. Firstly, there was heterogeneity across studies in terms of patient populations, surgical indications, imaging modalities, and outcome measures, which limits direct comparability. Second, while five of the six studies were RCTs, one was a single-arm phase I trial, and another was a non-randomized comparative cohort, introducing a moderate risk of bias. Third, long-term outcomes such as overall survival and quality-of-life metrics were not consistently reported across studies. Finally, the reconstructive component, although clinically significant, was less represented in high-level trials compared to neurosurgical contexts, underscoring an evidence gap in integrated multidisciplinary procedures.

Future Directions

This review highlights several important avenues for future research. Large-scale RCTs specifically evaluating intraoperative imaging in reconstructive or craniofacial procedures are needed to validate its broader applicability. Comparative studies across different imaging modalities (e.g., iMRI vs. iUS) would help refine modality-specific guidelines based on procedural complexity and anatomical region [18]. Economic evaluations assessing the cost-effectiveness of high-end systems like iMRI or machine vision are also warranted to guide institutional investment. Furthermore, the integration of artificial intelligence and augmented reality with intraoperative imaging represents an exciting frontier that could further enhance real-time decision-making and personalized surgery.

## Conclusions

This systematic review affirms that intraoperative imaging significantly enhances surgical precision, safety, and outcomes in combined neurosurgical and reconstructive procedures. The adoption of modalities such as iMRI, iUS, and fluoroscopy has demonstrable benefits in terms of extent of resection, complication reduction, and operative efficiency. These findings advocate for the broader clinical integration of intraoperative imaging, especially in multidisciplinary surgical settings. Future research should aim to expand evidence related to reconstructive domains and explore emerging technologies to optimize patient-centered surgical care.
